# Stimulatory Effects of Gamma Irradiation on Phytochemical Properties, Mitotic Behaviour, and Nutritional Composition of Sainfoin (*Onobrychis viciifolia* Scop.)

This article has been retracted.

**DOI:** 10.1155/2014/854093

**Published:** 2014-07-23

**Authors:** Sadegh Mohajer, Rosna Mat Taha, Ma Ma Lay, Arash Khorasani Esmaeili, Mahsa Khalili

**Affiliations:** ^1^Institute of Biological Sciences, Faculty of Science, University of Malaya, 50603 Kuala Lumpur, Malaysia; ^2^Department of Analytical Chemistry, Chemistry and Chemical Engineering Research Center, Tehran 14968-13151, Iran

## Abstract

Sainfoin (*Onobrychis viciifolia* Scop. Syn. *Onobrychis sativa* L.) is a bloat-safe forage crop with high levels of tannins, which is renowned for its medicinal qualities in grazing animals. Mutagenesis technique was applied to investigate the influence of gamma irradiation at 30, 60, 90, and 120 Gy on mitotic behavior, *in vitro* growth factors, phytochemical and nutritional constituents of sainfoin. Although a percentage of plant necrosis and non-growing seed were enhanced by irradiation increment, the germination speed was significantly decreased. It was observed that gamma irradiated seeds had higher value of crude protein and dry matter digestibility compared to control seeds. Toxicity of copper was reduced in sainfoin irradiated seeds at different doses of gamma rays. Anthocyanin content also decreased in inverse proportion to irradiation intensity. Accumulation of phenolic and flavonoid compounds was enhanced by gamma irradiation exposure in leaf cells. HPLC profiles differed in peak areas of the two important alkaloids, Berberine and Sanguinarine, in 120 Gy irradiated seeds compared to control seeds. There were positive correlations between irradiation dose and some abnormality divisions such as laggard chromosome, micronucleus, binucleated cells, chromosome bridge, and cytomixis. In reality, radiocytological evaluation was proven to be essential in deducing the effectiveness of gamma irradiation to induce somaclonal variation in sainfoin.

## 1. Introduction

Domestic animals feed on the fundamental nutrients comprising energy, protein, amino acids (macronutrients), minerals, vitamins, and other micronutrients. Sainfoin is a safe-bloating fodder crop which contains excessive protein. It is used for cattle, sheep, deer, and elk either as fodder feeding or as a grain concentrate. Grain concentrates are generally including a high intensity of nutrients and elevated degree of edible nutrients with low crude fibre substance (less than 18% of the dry matter).

Genetic variability is the most significant requirement for crop effective development with variant selections. In this respect, genetic variability can occur through the hybridization process, recombination, mutation, and selection. Natural selection has been exhausted in the sainfoin, which was not so productive [1]. Generated mutation is a reliable option for the sainfoin diversity which revives and redevelops in the variability.

Irradiation has been utilized effectively to cause suitable mutations for plant breeding improvement [2]. Many researchers have mentioned somaclonal differences for crop development by physical mutagens in particular, gamma irradiation. Gamma sources are exploited to irradiate varied plant components, such as seed, flower, anther, pollen grain, and single cell. Gamma irradiation mostly affects the plant growth by variation in production through cytology, biochemistry, physiology, and morphogenetic of the cells [3].

Various doses of gamma irradiation generate unrestricted radicals, which may induce unfavorable or useful components in plant cells. Some studies observed preventive effects in greater exposure of gamma rays, while lower exposures were occasionally more stimulating [4, 5]. In addition, the lower intensity of mutagenic treatment could improve the biochemical components, which has been consumed for enhancement of economical traits [2].

Mokobia and Anomohanran [6] realized that gamma irradiation was very notable not only for medical sterilization but also for seed nutritional maintenance. Moreover, the positive effects of gamma irradiation were indicated to raise the flavonoid, alkaloid, phenolic compound, and antioxidant activity [7]. Chlorophyll mutation is also one of the most dependable indicators to assess the genetic influences of mutagenic treatments. Impact of *γ*-irradiation could enhance seed quality traits, such as crude protein and digestibility, which are important in grain concentrate [8].

The present study was designed to observe the effects of gamma irradiation intensities on seed growing stages, investigate the feasibility of gamma irradiation to improve the phenolic compound, flavonoid, alkaloid, anthocyanin, and other pigments, evaluate the effect and role of gamma irradiation on seed nutritional improvement, and determine the appropriate irradiation dose for somaclonal variation which is subsequently verified by cytological assessment.

## 2. Materials and Methods

### 2.1. Plant Materials and Gamma Treatment

Gamma treatment was obtained from 60 Cobalt, 0026 Pool Irradiator with isotope model, while the dose rate was 0.0627 Gy/second. Seeds of* Onobrychis viciifolia* were exposed to 4 different levels of 30, 60, 90, and 120 Gy. Non-irradiated seeds were also used as the control treatment.

Seeds were sterilized after gamma irradiation. Sterilized seeds were germinated on MS medium supplemented with 30 g/L sucrose and 7.8 g/L agar (at pH 5.8). Cultures were maintained at 25 ± 2°C under 70% humidity and 16 h light photoperiod provided by fluorescent lamps [9].

### 2.2. Growth Parameters

In order to determine the growth rate of cells, control and irradiated seeds were assessed based on their growing stages after 2 months. Speed of germination was calculated based on the following formula during the first week [10]:

(1) Speed  of  germination =X1Y1+X2−X1Y2+⋯+Xn−Xn−1Yn

(where *X*_1_, *X*_2_, and *X*_*n*_ were number of seeds germinated of the first, second, and *n*th day, resp. *Y*_1_, *Y*_2_, and *Y*_*n*_ were number of sowing days of the first, second, and *n*th count, resp.).

### 2.3. Measurement of Pigment Contents

After germination, two grams of fresh leaves was homogenized using chilled mortar containing 10 mL of methanol (80% v/v) and some MgCO_3_. Sample extract was collected and filtered using the Buchner funnel through Whatman filter paper no. 5. Extract volume was topped up to 50 mL with methanol (80% v/v). Samples were centrifuged at 3000 rpm for 5 minutes. Adsorption values were measured at 666 nm, 653 nm, and 470 nm using Shimadzu spectrophotometer. Contents of chlorophyll a (C_a_), chlorophyll b (C_b_), and total carotenoid were assessed based on the modified formulae by Lichtenthaler and Wellburn [11] based on micro g/g FW:

(2) Ca=15.65A666−7.340A653,Cb=27.05A653−11.21A666,Cx+c=1000A470−2.860Ca−(129.2Cb/245).

For measurement of anthocyanin content, 0.1 g of samples was grounded in 3 mL of acidified methanol (99 : 1 of methanol : HCl). Samples were then centrifuged at 12000 rpm for 20 minutes and the supernatant was kept in the dark, at 4°C for 24 h. Absorbance was recorded at 550 nm, and anthocyanin content was calculated based on an extinction coefficient of 33000/Mol cm [12].

### 2.4. Total Flavonoid Determination

Aluminium chloride colorimetric method [13] was used for the evaluation of flavonoid in fresh leaves of* in vitro* grown plants. Each methanol extract (0.5 mL of 1 : 10 g/mL) was separately mixed with 1.5 mL methanol, 0.1 mL 10% aluminum chloride, 0.1 mL 1 M potassium acetate, and 2.8 mL distilled water. Extracts were kept at room temperature for 30 min. Absorbance of mixed reaction was measured at 415 nm using Shimadzu spectrophotometer. Calibration curve was prepared by measuring the methanol quercetin solutions at 20 to 100 *μ*g/mL concentrations.

### 2.5. Total Phenolic Compounds

Total phenolic compounds were determined by Folin Ciocalteu reagent in fresh leaves [14]. Each methanol diluted extract (0.5 mL of 1 : 10 g/mL) was mixed with the Folin Ciocalteu reagent (5 mL, 1 : 10 dilution using distilled water) and aqueous Na_2_CO_3_ (4 mL, 1 M). The mixtures were retained for 15 min. Total phenols were determined by absorption measurement at 765 nm using Shimadzu spectrophotometer. A standard curve was prepared by using the methanol Gallic acid solutions at 20 to 100 *μ*g/mL concentrations.

### 2.6. HPLC-UV Analysis

Standard solution of Sanguinarine and Berberine was purchased from Sigma (USA). Chemical structures of alkaloids are shown in Figure 2. HPLC system (Knauer K-2600) coupled with UV detector was used for quantitative determination of two alkaloids in both non-irradiated (control) and 120 Gy irradiated seed powder. UV detector was set at the wavelength of 280 nm and area was used for quantification. Chromatographic separation was carried out on Kromasil C18 analytical column (5 *μ*m, 250 mm × 4.6 mm) at 30°C. Linear gradient elution of *A* (100% acetonitrile) and *B* (0.1% phosphoric acid aqueous solution) was used. Time program for multistep gradient was initially 27% (*A*), 0−5 min keeping 27% (*A*), 5−17 min linear gradient to 54% (*A*), 17−20 min from 54% to 75% (*A*), 20−25 min from 75% to 80% (*A*), 25−35 min keeping 80% (*A*), 35−40 min linear gradient to 27% (*A*), and keeping 27% (*A*) at 40−45 min. The flow rate was 0.8 mL/min and injection volume was 5 *μ*L. Calibration curves were drawn based on the reference (standards) areas against their respective concentrations.

### 2.7. Quality Traits Assessment

A percentage of crude fibre (CF), crude protein (CP), dry matter digestibility (DMD), water soluble carbohydrates (WSC), acid detergent fibre (ADF), neutral detergent fibre (NDF), and ash of both non-irradiated (control) and irradiated samples were determined in dry seed powder using near infrared radiation (NIR) spectroscopy. After calibration, percentages of quality traits were calculated using the method by Jafari et al. [15].

### 2.8. Atomic Absorption Spectrometry

Seed powder was also analyzed for different elements of Mn, Cu, Ca, P, and N (based on the ratio of irradiated samples to control) according to the methods described by AOAC [16] using atomic absorption spectrometry (Young Lin AAS-8020).

### 2.9. Cytometric Parameters

Permanent slides of meristematic root cells were prepared based on the methods described by Conger and Fairchild [17] from irradiated and non-irradiated* in vitro *grown plants. Slides were evaluated using a light microscope (Zeiss Axioscope, Germany) connected to a Sony Video Camera. Image analyzer was used for the assessment of mitotic index, cell and nuclear areas. Various abnormality divisions were also estimated based on the chromosome disorder.

### 2.10. Statistical Analysis

The frequency of mitosis was determined by counting the number of dividing cells in total 150 of the cells. Results were expressed as mean ± standard error. The effects of treatments were tested by variance analysis and differences between samples were determined by Duncan's multirange test at *P* < 0.05 using SAS 9.2 software.

## 3. Results

While irradiated and non-irradiated seeds were germinated simultaneously after 2-3 days of sowing, germination rate was only indicated to be 100% in the control seeds (Table 1). A percentage of necrosis and non-growing seeds were found to increase gradually when the seeds were exposed to gamma irradiation. Germination speed was revealed to decrease with an increment of gamma irradiation intensities. Approximately, the highest shooting percentage was observed in control seeds after one month with 82.11%. Maximum shoot number was observed when the seeds were not treated with the gamma irradiation (Table 1).

Gamma irradiation intensities were indicated to reduce the anthocyanin content significantly in* in vitro* grown plants. Fresh leaf extractions exhibited an initial enhancement of chlorophyll content. In this regard, chlorophylls a and b had the highest amount at 30 Gy and 60 Gy of gamma irradiation, respectively. Carotenoid content also rose gradually with the increasing of irradiation intensity up to 90 Gy (Table 2). Carotenoid plays an important role in light protection of chlorophyll from photo-oxidative damage. Thus, the carotenoid content reduction could have a serious impact on photosynthetic and chlorophyll pigments.

Flavonoid content derived extracts confirmed the highest amount in 90 Gy intensity of gamma irradiation in terms of quercetin equivalent (*y* = 0.148*x* − 0.0242, *R* ^2^ = 0.991). Total phenolic contents measured by Folin Ciocalteu reagent were assessed in terms of Gallic acid equivalent (*y* = 0.1077*x* − 0.0377, *R* ^2^ = 0.979). Remarkable increase was observed in phenolic contents of 90 Gy irradiated leaf extract compared to non-irradiated (control) extract (Figure 1).

Two alkaloid compounds (Berberine and Sanguinarine) were also measured in both 120 Gy irradiated and non-irradiated seed powder (Figure 2). Good linearity (*R* ^2^ = 0.995) was achieved in both calibration curves of the alkaloids. Sanguinarine content decreased when the seeds were subjected to 120 Gy intensity of gamma irradiation, from 0.000121% to 0.000112%. Furthermore, Berberine content was improved when the seeds were exposed to gamma irradiation, from 0.000152% to 0.000203%. Sanguinarine and Berberine of irradiated seeds were detected after control seeds in HPLC chromatogram due to the different dilutions used (Figure 3).

Seed quality and nutritional value were directly correlated with crude protein (CP) and dry matter digestibility (DMD). Nutritional quality had also an inverse relation with acid detergent fibre (ADF) and crude fibre (CF). A percentage of CP and DMD were significantly different in gamma irradiated seeds compared to control seeds. The highest CP (34.20%) and DMD (94.53%) were observed when the seeds were exposed to 30 Gy and 120 Gy irradiation, respectively. In addition, the exposure of gamma irradiation had the positive effect in seed quality improvement with reduction of CF percentage. Percentage of water-soluble carbohydrates (WSC) went up with increasing gamma irradiation intensity. On the other hand, percentage of acid detergent fibre (ADF) was gradually decreased with enhancement of gamma irradiation gray. No significant difference was indicated in terms of the ash percentage between gamma treated seeds and control seeds (Table 3).

Ratio of trace metals (Mn and Cu) and macronutrients (Ca, P, and N) in irradiated seeds to non-irradiated seeds was determined using atomic absorption spectrophotometry (AAS) as shown in Figure 4. Exposure to 30 Gy gamma irradiation had positive effects on improving the N contents. In reality, the novel efficiency of gamma exposure was observed in the amount of P. In contrast, ratio of Ca, Mn, and Cu were found to decrease with gamma irradiation (Figure 4).

Mitotic index (MI) was used as an indicator to describe the cell activity and proliferation. It was observed that MI of root meristematic cells increased from 26.51% to 34.53% when the seeds were exposed to 60 Gy of gamma irradiation. The majority of the cells were found to be in prophase stage in both* in vitro* irradiated and non-irradiated samples (Table 4 and Figure 5). In general, mean cell and nuclear areas were significantly increased in the treated plants compared to control plants. The highest nuclear and cell areas were noted at the lowest intensity (30 Gy) of gamma irradiation with 188.44 *μ*m^2^ and 875.40 *μ*m^2^, respectively (Table 5).

Although, the most of the cell cycle segregation displayed regular mitosis in both control and irradiated cells, some mitotic abnormalities were also observed. Effect of gamma irradiation intensities on mitotic irregularities was assessed in terms of the chromosome laggards and bridge, binucleated cells, chromosome fragmented, asynchronous nuclei, cytomixis, desynapsis, and micronucleus (Table 6 and Figure 5). Gamma irradiation exposure by 120 Gy exhibited higher mitotic irregularities percentage compared to other specimens. Cytomixis, desynapsis, and chromosome fragmented were only observed in the irradiated cell division. Gamma irradiation also increased the occurrence of binucleated cells. In addition, the percentage of the chromosome laggard/bridge was observed to rise with an increment of gamma irradiation intensity (Table 6 and Figure 5).

## 4. Discussion

Gamma rays belong to ionizing radiation that reacts with atoms or molecules to generate free radicals in cells. These radicals can transfigure essential constituent of plant cells. Some studies have been accomplished to show the influence distinctively in biochemistry, physiology and morphology by different doses of gamma irradiation[18]. The variety improvement through radiation needs an essential study to distinguish whether/how it can affect each species. So, the positive and negative consequences of gamma intensities were evaluated in this paper. Although, gamma intensities had the negative influence on plant growth, the positive effects were observed at 60 and 90 Gy in phytochemical properties of sainfoin. It has been found that plant growth was stimulated at 10 Gy in* Citrus sinensis* and inhibition occurred at radiation intensities more than 10 Gy [19]. Correspondingly, Norfadzrin et al. [20] observed that the high gamma ray doses had a negative influence on the morphological traits of tomato and okra seedlings obtained from irradiated seeds. Results of 120 Gy were not significantly different compared to 90 Gy in nutritional composition of sainfoin. Some researchers have shown that the higher exposures of gamma radiation were usually inhibitory by reduction of mitotic activity, whereas low doses of gamma irradiation could be used as safer and more stimulatory tools to improve variations [21, 22]. Some scientists stated that low doses of irradiation stimulate growing by changing the hormonal influence in the plant cells. In addition, low intensities improved the antioxidative capability of cells to dominate stress factors such as temperature in* in vivo* growth culture [23]. As a whole, gamma irradiation considerably reduced shoot formation and rate of germination as compared with control treatment, which is presented in Table 1. Growth blockage caused through the high amount of irradiation resulted in the cell cycle arrest at the G2/M phase during somatic cell division or genome damages [24].

Biochemical variations were observed in chlorophyll, carotenoid, and anthocyanin contents of irradiated and non-irradiated leaves after four weeks of this study. Strid et al. [25] indicated that gamma irradiation can damage pigments with simultaneous loss of photosynthetic ability which was not adapted in our outcomes of chlorophylls a and b. Respectively, low intensities of gamma irradiation were more effective to produce the chlorophyll mutations in sainfoin. Observations of this research were in accordance with those acquired by Rascio et al. [26], Osama [27], and Rejili et al. [28]. They found chlorophyll improvement after applying different mutagenic treatments such as E.M.S, sodium azide, and gamma rays. Apparently, the mutation of chlorophyll b was moderately less than chlorophyll a through gamma irradiation. It was as a result of more selective damage of decadence biosynthesis in chlorophyll (a) precursors. It was revealed that the higher amount of irradiation led to anthocyanin degradation. This result was not in agreement with those stated by Abo-EI-Seoud et al. [29], since they realized that the capability of 40 Gy increased the anthocyanin content.

Phytochemical properties such as flavonoid, phenol, and alkaloid have an indirect effect on fodder quality. Phytochemical analysis showed changes in the status of phenol content, flavonoid content (in leaves), and alkaloid presence (in seeds) in the sainfoin as a result of irradiation treatment. Irradiation may cause oxidative damage and impair the flavor in plants. However, the effective action and radio-stable nature of antioxidants can protect the chemical oxidation of biomolecules in irradiated plants. Similar to our observations, the ability of gamma irradiation has been also confirmed to increase the phenolic acids of plant metabolites in soybean samples treated with gamma irradiation at levels ranging from 50 to 150 Gy [30].

Grain concentrates are utilized by many ruminant production systems. Grain concentrates may develop a high amount of diets for milk and meat production (over 30% and 70%, resp.). Sainfoin seed concentrates can also provide high crude protein and dry matter digestibility, consisting of a mixture of vegetable proteins, urea, important vitamins, and minerals. The highest proportion of crude protein was verified at 30 Gy treated seeds compared to control seeds. Dhopte et al. [31] also indicated significant differences in protein percentage of chickpea seeds in various intensities. Therefore, there is a high possibility to improve the crude protein in some kinds of genotypes by utilizing gamma ray.

Based on previous research [32], there are significant and direct relations between seed and forage quality in sainfoin. In this regard, nutritional composition of seed was evaluated after irradiation. Some parameters like crude protein, crude fibre, and digestibility were analyzed, which have a direct effect on either grain concentrate or hay quality. Development of the defensive systems is the most significant reaction of plant cells to gamma irradiation. The CP was calculated for the significant difference between control seeds and irradiated seeds, which was in conformity with the results obtained by Lawal et al. [33]. Increasing the amount of crude protein has been used as a protective mechanism against the damages of gamma irradiation [34]. Consistent with assessment results of the present study, Osunde [35] reported no significant difference in the crude fibre content. Unlike our evaluation, Štajner et al. [36] implicated that gamma treatment did not induce significant increment in water soluble components such as minerals, nitrogenous constituents, and sugars. The ash percentage remained unaffected by irradiation processing, which was associated with mineral content in sainfoin. However, the ash content was lower in the control seeds.

A mutation in availability of Ca is not probably the main objective of a study, since the amount involved in metabolic processes is usually small compared to those present in the soil. Likewise, gamma irradiation increased the amount of P and N released in the soil after 2 weeks of incubation, which was observed in the studied sainfoin seeds [37]. Nitrogen and P are constituents of both the living and dead plants in the soil. Cells death and the subsequent degradation can occur due to the ionization effect of gamma ray on living organisms, which results in increasing the P and N release rate.

Despite the fact that a number of mutant plants are identified in M_2_ generation, there is convincing evidence of correlation between M_1_ treated plant and mutation frequency in M_2_ induced by ionizing radiations. That is why a quantitative determination of M_1_ destruction can be an inevitable step in mutation breeding, especially for plant species such as sainfoin that has not been studied extensively for crop improvement. The assessments of the mitotic cycle in shoot or root meristem cells offered a reliable test to determine the influence of the mutagens in M_1_ [38]. The evaluation of chromosome configuration by cytological analysis provides a direct vision of induced chromosomal rearrangements. In this regard, the frequency and spectrum of chromosomal aberrations were analyzed at anaphase in this study. The induction of cytological disturbances is important in the mitotic division, since genome damage is handed over to the next generation [39]. Increment of nuclear and cell areas confirmed that various mutagens had different mutagenic potential. In the present investigation, the mutagenic treatments exhibited higher types of aberrations in sainfoin. Along this line, abnormality division variations have been widely evaluated to understand the mechanisms of induced chromosomal damage. A higher proportion of chromosomal aberrations were indicated to chromosomes stickiness, which might have been enhanced due to depolymerization of nucleic acid and partial dissociation of the nucleoproteins [40]. Laggard chromosome generally leads to micronuclei formation [41]. Micronuclei were induced when the laggard chromosomes fail to reach the poles in time of the telophase [42]. Chromosomes bridges could also occur through breaks in two chromosomes followed by the union of centric fragments [43]. Ultimately, more abnormalities accumulated which cause nonviable gametes and plant fertility reduction.

## Figures and Tables

**Figure 1:** Effect of gamma irradiation on flavonoid and phenol compounds of* in vitro* leaves. The means of the samples with the same small letters were not significantly different as per Duncan's multirange test at *P* < 0.05.

**Figure 2:** Chemical structures of two alkaloids identified in* Onobrychis viciifolia*.

**Figure 3:** HPLC chromatograms of control and *γ*-irradiated seeds (120 Gy) according to standard mixture. Retention time has been adjusted based on the centesimal unit in this experiment.

**Figure 4:** Ratio of element contents in gamma-irradiated seeds to non-irradiated (control) sample.

**Figure 5:** Root meristem cells of* O. viciifolia *showing normal and abnormal mitosis. (a) prophase, (b) metaphase, (c) anaphase, (d) telophase, (e) fragmented chromosomes, (f) micronucleus, (g) asynchronous nucleus, (h) binucleated cells, and (i) cytomixis. Bars = 10 *μ*m.

**Table 1:** Effect of gamma irradiation on growth stages of *Onobrychis viciifolia *seeds after 4 weeks.

Gamma irradiation (Gy)	Non-growing (%)	Necrosis (%)	Shooting (%)	Mean number of shoots	Germination speed
Control	0.00^c^	17.89^c^ ± 2.24	82.11^a^ ± 3.42	3.55^a^ ± 0.15	20.41^a^ ± 1.52
30	5.56^b^ ± 0.85	22.52^bc^ ± 2.25	72.22^ab^ ± 3.36	2.46^b^ ± 0.18	18.24^a^ ± 1.84
60	7.26^ab^ ± 0.64	32.38^b^ ± 2.36	60.18^bc^ ± 2.18	2.04^b^ ± 0.24	17.01^ab^ ± 1.31
90	9.54^a^ ± 1.17	40.49^ab^ ± 3.32	50.07^c^ ± 2.32	2.75^b^ ± 0.15	15.27^b^ ± 1.33
120	10.15^a^ ± 1.12	48.01^a^ ± 2.41	42.23^c^ ± 2.38	2.84^b^ ± 0.16	14.37^b^ ± 1.65

The means of samples with the same small letters were not significantly different as per Duncan's multirange test at *P* < 0.05.

**Table 2:** Effect of gamma irradiation on chlorophyll, carotenoid, and anthocyanin contents of *in vitro* leaves.

Gamma irradiation (Gy)	Control	30	60	90	120
Chlorophyll a (*μ*g/g FW)	15.86^b^ ± 0.24	19.45^a^ ± 1.01	18.04^a^ ± 0.64	17.74^a^ ± 1.14	16.59^ab^ ± 1.06
Chlorophyll b (*μ*g/g FW)	10.54^b^ ± 0.33	12.65^a^ ± 0.94	13.66^a^ ± 1.06	12.68^a^ ± 0.92	11.13^ab^ ± 0.71
Carotenoid (mg/g FW)	1.59^b^ ± 0.07	2.22^a^ ± 0.08	2.19^a^ ± 0.05	2.14^a^ ± 0.05	1.84^b^ ± 0.03
Anthocyanin (mMol/g FW)	14.8^a^ ± 0.86	14.5^a^ ± 0.96	10.6^b^ ± 0.85	10.9^b^ ± 1.07	7.88^c^ ± 0.72

The means of the samples with the same small letters were not significantly different as per Duncan's multirange test at *P* < 0.05.

**Table 3:** Mean comparison of nutritional traits among irradiated and non-irradiated *O. viciifolia* seeds.

Gamma irradiation (Gy)	CP %	DMD %	WSC %	ADF %	NDF %	ASH %	CF %
Control	32.24^b^ ± 2.1	89.68^b^ ± 2.3	34.31^a^ ± 1.2	11.39^a^ ± 0.8	9.99^b^ ± 0.6	5.35^a^ ± 0.2	23.35^a^ ± 1.6
30	34.80^a^ ± 2.2	93.35^a^ ± 2.2	34.40^a^ ± 1.4	8.43^b^ ± 0.9	10.78^b^ ± 0.8	5.87^a^ ± 0.4	23.63^a^ ± 1.3
60	33.53^a^ ± 1.5	92.13^a^ ± 1.8	34.90^a^ ± 1.1	9.81^b^ ± 0.7	12.35^a^ ± 0.6	5.65^a^ ± 0.5	23.52^a^ ± 1.4
90	33.13^a^ ± 1.3	92.22^a^ ± 1.8	34.91^a^ ± 0.9	9.41^b^ ± 0.7	9.92^b^ ± 0.6	5.73^a^ ± 0.5	23.06^a^ ± 1.4
120	34.02^a^ ± 2.3	94.53^a^ ± 2.1	35.42^a^ ± 1.2	7.17^b^ ± 0.8	9.83^b^ ± 0.7	5.91^a^ ± 0.4	22.87^a^ ± 1.8

The means of samples with the same small letters were not significantly different as per Duncan's multirange test at *P* < 0.05.

Crude protein (CP), crude fibre (CF), acid detergent fibre (ADF), dry matter digestibility (DMD), water soluble carbohydrates (WSC), and neutral detergent fibre (NDF).

**Table 4:** Effect of gamma irradiation on mitotic behavior of *Onobrychis viciifolia* in* in vitro *growth culture.

Gamma irradiation (Gy)	Mitosis stages					Mitotic index (MI)
	Interphase	Prophase	Metaphase	Anaphase	Telophase	
Control	73.47^a^ ± 2.21	20.33^b^ ± 2.19	3.82^b^ ± 0.24	1.49^a^ ± 0.21	0.97^b^ ± 0.09	26.51^b^ ± 1.65
30	63.97^b^ ± 2.10	25.41^a^ ± 2.24	5.58^a^ ± 0.12	2.11^a^ ± 0.11	2.38^a^ ± 0.12	35.07^a^ ± 1.74
60	65.29^b^ ± 2.24	24.24^a^ ± 2.28	6.13^a^ ± 0.14	2.42^a^ ± 0.14	2.02^a^ ± 0.18	34.53^a^ ± 1.57
90	65.55^b^ ± 2.16	22.06^b^ ± 2.34	7.57^a^ ± 0.17	2.35^a^ ± 0.39	2.24^a^ ± 0.15	34.32^a^ ± 1.66
120	67.15^b^ ± 2.13	21.30^b^ ± 2.24	7.32^a^ ± 0.17	2.06^a^ ± 0.51	2.13^a^ ± 0.12	32.82^b^ ± 1.63

The means of samples with the same small letters were not significantly different as per Duncan's multirange test at *P* < 0.05.

**Table 5:** Effect of gamma irradiation on cell and nuclear area of *Onobrychis viciifolia* in *in vitro *growth culture.

Gamma irradiation (Gy)	Nuclear (*μ*m^2^)	Cell (*μ*m^2^)	N/C
Control	141.25^b^ ± 7.9	668.72^b^ ± 15.2	0.21
30	188.44^a^ ± 6.3	875.40^a^ ± 24.4	0.22
60	182.63^a^ ± 8.4	782.69^a^ ± 20.1	0.23
90	186.41^a^ ± 6.6	802.81^a^ ± 18.2	0.23
120	183.86^a^ ± 5.3	829.60^a^ ± 18.4	0.22

The means of samples with the same small letters were not significantly different as per Duncan's multirange test at *P* < 0.05.

**Table 6:** Effect of gamma irradiation on mitotic aberrations of *Onobrychis viciifolia* in *in vitro* growth culture.

Gamma irradiation (Gy)	Cytomixis (%)	Fragmented (%)	Bridge/laggard (%)	Micronucleus (%)	Asynchronous nucleus (%)	Binucleated cells (%)	Desynapsis (%)
Control	0.00	0.00	0.42 ± 0.05	0.44 ± 0.04	0.40 ± 0.05	0.97 ± 0.08	0.00
30	2.78 ± 0.32	0.00	1.34 ± 0.11	0.58 ± 0.05	0.87 ± 0.10	1.14 ± 0.16	0.00
60	2.44 ± 0.25	0.67 ± 0.08	2.32 ± 0.14	0.54 ± 0.05	1.22 ± 0.13	1.32 ± 0.18	1.22 ± 0.15
90	1.94 ± 0.14	1.20 ± 0.10	1.23 ± 0.16	0.64 ± 0.05	0.67 ± 0.08	1.29 ± 0.18	1.94 ± 0.17
120	2.11 ± 0.22	2.14 ± 0.21	2.26 ± 0.18	1.06 ± 0.12	1.08 ± 0.18	2.18 ± 0.24	1.06 ± 0.13

## References

[1] Wani AA, Anis M (2001). Gamma rays induced bold seeded high yielding mutant in chickpea. *Mutation Breeding Newsletter*.

[2] Muthusamy A, Vasanth K, Jayabalan N (2003). Response of physiological and biochemical components in *Gossypium hirsutum* L. to mutagens. *Journal of Nuclear Agriculture and Biology*.

[3] Rahimi MM, Bahrani A (2011). Effect of gamma irradiation on qualitative and quantitative characteristics of Canola (*Brassica napus* L.). *Middle-East Journal of Scientific Research*.

[4] Radhadevi DS, Nayar NK (1996). Gamma rays induced fruit character variations in Nendran, a variety of banana (*Musa paradasiaca* L.). *Geobios*.

[5] Thapa CB (1999). Effect of acute exposure of gamma rays on seed germination of *Pinuskesiya* Gord and *P. wallichiana*. *Botanica Orientalis*.

[6] Mokobia CE, Anomohanran O (2005). The effect of gamma irradiation on the germination and growth of certain Nigerian agricultural crops. *Journal of Radiological Protection*.

[7] Kim JK, Jo C, Hwang HJ, Park HJ, Kim YJ, Byun MW (2006). Color improvement by irradiation of *Curcuma aromatica* extract for industrial application. *Radiation Physics and Chemistry*.

[8] Yami A (2008). *Nutrition and Feeding of Sheep and Goats*.

[9] Mohajer S, Taha RM, Khorasani A, Yaacob JS (2012). Induction of different types of callus and somatic embryogenesis in various explants of Sainfoin (*Onobrychis sativa*). *Australian Journal of Crop Science*.

[10] Maguire JD (1962). Speed of germination—aid in selection and evaluation for seedling emergence and vigor. *Crop Science*.

[11] Lichtenthaler HK, Wellburn AR (1985). Determination of total carotenoids and chlorophylls A and B of leaf in different solvents. *Biochemical Society Transactions*.

[12] Sarghein SH, Carapetian J, Khara J (2008). Effects of UV radiation on photosynthetic pigments and UV absorption compounds in *Capsicum longum* L.. *International Journal of Botany*.

[13] Chang C, Yang M, Wen H, Chern J (2002). Estimation of total flavonoid content in propolis by two complementary colometric methods. *Journal of Food and Drug Analysis*.

[14] McDonald S, Prenzler PD, Antolovich M, Robards K (2001). Phenolic content and antioxidant activity of olive extracts. *Food Chemistry*.

[15] Jafari AA, Connolly V, Frolich A, Walsh EK (2003). A note on estimation of quality parameters in perennial ryegrass by near infrared reflectance spectroscopy. *Irish Journal of Agricultural and Food Research*.

[16] AOAC (2003). *Official Methods of Analysis of the Association of Official’s Analytical Chemists*.

[17] Conger AD, Fairchild LM (1953). A quick-freeze method for making smear slides permanent. *Stain Technology*.

[18] Wi SG, Chung BY, Kim JH (2005). Ultrastructural changes of cell organelles in *Arabidopsis* stems after gamma irradation. *Journal of Plant Biology*.

[19] Ling APK, Chia JY, Hussein S, Harun AR (2008). Physiological responses of *Citrus sinensis* to gamma irradiation. *World Applied Sciences Journal*.

[20] Norfadzrin F, Ahmed OH, Shaharudin S, Rahman DA (2007). Apreliminary study on pigments and antioxidant machineries of red pepper (*Capsicum annuum* L.) seedlings from gamma-irradiated seeds. *Journal of Plant Biology*.

[21] Kumari R, Singh Y (1996). Effect of gamma rays and EMS on seed germination and plant survival of *Pisum sativum* L. and *Lens culinaris*. *Medicine Neo Botanica*.

[22] Khalil SJ, Rehman S, Afridi K, Jan MT (1986). Damage induced by gamma irradiation in morphological and chemical characteristics of barley. *Sarhad Journal of Agriculture*.

[23] Moghaddam SS, Jaafar H, Ibrahim R, Rahmat A, Aziz MA, Philip E (2011). Effects of acute gamma irradiation on physiological traits and flavonoid accumulation of *Centella asiatica*. *Molecules*.

[24] Preuss SB, Britt AB (2003). A DNA-damage-induced cell cycle checkpoint in arabidopsis. *Genetics*.

[25] Strid A, Chow WS, Anderson JM (1990). Effects of supplementary ultraviolet-B radiation on photosynthesis in *Pisum sativum*. *Biochimica et Biophysica Acta: Bioenergetics*.

[26] Rascio A, Russo M, Mazzucco L, Platani C, Nicastro G, Di Fonzo N (2001). Enhanced osmotolerance of a wheat mutant selected for potassium accumulation. *Plant Science*.

[27] Osama MS (2002). *Molecular genetic studies onirradiated wheat plants [Ph.D. thesis]*.

[28] Rejili M, Telahigue D, Lachiheb B, Mrabet A, Ferchichi A (2008). Impact of gamma radiation and salinity on growth and K^+^/Na^+^ balance in two populations of *Medicago sativa* (L.) cultivar Gabès. *Progress in Natural Science*.

[29] Abo-EI-Seoud MA, Hashim MF, Farid AM Combined Effect of Gamma radiation and potassium fertilization on growth and coloring matter contents of roselle (*Hibiscus Sabdariffa* L.).

[30] Variyar PS, Limaye A, Sharma A (2004). Radiation-induced enhancement of antioxidant contents of soybean (*Glycine max* Merrill). *Journal of Agricultural and Food Chemistry*.

[31] Dhopte AM, Thombre PG, Patil VK (1974). Physiological studies of radiation induced mutants in gram. *Journal of Tropical Agriculture*.

[32] Mohajer S, Jafari AA, Taha RM (2011). Studies on seed & forage yield in 10 populations of sainfoin (*Onobrychis sativa*) grown as spaced plants & swards. *Journal of Food, Agriculture & Environment*.

[33] Lawal AO, Akueche EC, Anjorin ST (2011). Effects of gamma irradiation on the sprouting, nutritional and phytochemical composition of Meccakusha yam tubers in Abuja, Nigeria. *Journal of Agriculture and Biological Sciences*.

[34] Al-Rumaih MM (2008). Influence of ionizing radiation on antioxidant enzymes in three species of *Trigonella*. *American Journal of Environmental Sciences*.

[35] Osunde ZD (2008). Minimising Postharvest losses in Yam ( Dioscorea spp.). *Treatment and Techniques: In: Using Food Science and Technology: In Improving Nutritional and Promote National Development*.

[36] Štajner D, Milošević M, Popović BM (2007). Irradiation effects on phenolic content, lipid and protein oxidation and scavenger ability of soybean seeds. *International Journal of Molecular Sciences*.

[37] Eno F, Popenoe H (1963). The effect of gamma radiation on the availability of nitrogen and phosphorus in soil. *Division S-3-Soil Microbiology*.

[38] Gaul H (1977). *Mutagen Effects in the First Generation after Seed Treatment*.

[39] Kumar G, Rai P (2007). Comparative genotoxic potential of mercury and cadmium in soybean. *Turkish Journal of Biology*.

[40] Kumar G, Kesarwani S, Sharma V (2003). Clastogenic effect of individual and combined treatment of Gamma rays and EMS in *Lens culinary*. *Journal of Cytology and Genetics*.

[41] Kumar G, Rai P (2006). Partial genome elimination through micronuclei in soybean (*Glycine max*). *National Academy of Science Letters*.

[42] Utsunomiya KS, Bione NCP, Pagliarini MS (2002). How many different kinds of meiotic abnormalities could be found in a unique endogamous maize plant?. *Cytologia*.

[43] Shreekrishna V (2006). Cytological Abnormalities in Amaranthus paniculatus treated with Ethyl Methyl sulphonate. *Journal of Cytology and Genetics*.

